RETRACTED

# Anterior Cruciate Ligament Reconstruction with Hybrid Graft versus Autograft: A Systematic Review and Meta-Analysis

**DOI:** 10.1155/2021/7562649

**Published:** 2021-10-06

**Authors:** Ning Li, Xiali Xue, Huan Tu, Ming Zhang, Chengqi He

**Affiliations:** ^1^Center of Rehabilitation Medicine, West China Hospital, Sichuan University, Chengdu, Sichuan, China; ^2^Department of Biomedical Engineering, The Hong Kong Polytechnic University, Hong Kong, China; ^3^Institute for Disaster Management and Reconstruction, Sichuan University-The Hong Kong Polytechnic University, Chengdu, Sichuan, China; ^4^Institute of Sports Medicine and Health, Chengdu Sport University, Chengdu, Sichuan, China

## Abstract

**Background:**

The standard surgical treatment for ACL tear is ACL reconstruction. There is a debate of a choice between autograft or hybrid graft for treating ACL reconstruction. The purpose of this paper is to compare both case scenarios.

**Methods:**

A lot of libraries were searched like PubMed, Cochrane, and EMBASE Library for clinical trials which were then compared and analyzed via meta-analysis. The systematic review and meta-analysis were performed as per PRISMA guidelines, and RevMan software was used to perform the meta-analysis.

**Results:**

We analyzed 6 studies where patients of both autograft and hybrid graft were studied. The study outcomes, graft failures, graft diameters, reoperations, and so on were compared via forest plot and funnel plot. No significant difference was noted in both cases.

**Conclusions:**

In this meta-analysis, the performance of both autograft and hybrid graft was similar. Though the diameters were larger in hybrid, other factors also had an influence like graft failures, reoperations, and age at reconstruction which must be further investigated in detail.

## 1. Introduction

Anterior cruciate ligament reconstruction (ACL/ACLR) is one of the most recommended procedures by surgeons in case of sports injury. Every year more than 100,000 patients require ACL reconstruction (ACLR) in US. Even though due to better tendon, bone healing chances, autologous graft reconstruction is a popular choice. However, many evidences have shown that 8 mm autografts have no guarantee of good prognosis mainly in young patients [1, 2].

Knee ioint is comprised of multiple articulations which in turn is responsible for handling multiple physical activities and responding to loads. ACL is a ligament which connects femur to tibia and hence gets torn due to pivot movements leading to knee instability.

The main aim of the surgery is to recreate the anatomy of the ACL thus stabilizing the knee joint and hence preventing rupturing of the graft due to technical flaws in the procedures. This surgery is a treatment option for the young athletes or for those professionals who demand stability in the progressively degenerating knee conditions with long instabilities. This treatment resolves and fulfills the occupational demands for those who pursue sports as a profession [3–5].

RETRACTED

Commonly opted graft options are semitendinosus-gracilis autograft, various allografts, bone-patellar tendone-bone autograft, and distal quadriceps autograft [6, 7].

A very popular choice of graft is semitendinosus-gracilis autograft which has been proven in many research studies as it has shown high patient satisfaction, knee laxity, patient outcomes, and various other functionality tests when compared against autografts [1, 8, 9].

In this paper, we have performed a systematic review and meta-analysis on anterior cruciate ligament reconstruction with hybrid graft in comparison to autograft so as to analyze the risk benefit and success failure cases and get a comparative analysis of both treatments.

## 2. Methodology

### 2.1. Search Strategy

A search of data was performed using Ovid of Medline (1950 to May 2021), EMBASE (1974 to May 2021), AMED (1985 to May 2021), and CINAHL (1982 to May 2021) using MeSH terms in order to identify the papers of randomized and nonrandomized clinical trials thus successfully comparing the outcomes of hybrid graft versus autograft in anterior cruciate ligament reconstruction. The PRISMA for selecting the studies is shown in Figure 1. They key words used for searching the research studies were ‘‘anterior cruciate ligament reconstruction,” “surgery,” “ACL,” “ACLR,” “anterior cruciate ligament reconstruction,” “autograft,” “hybrid graft versus autograft,” “hybrid graft,” “surgery,” “sports injury,” “knee ligament surgery,” “orthopedic surgery,” and “ligament reconstruction.” More unpublished literatures were searched using the term “Anterior cruciate ligament reconstruction” from other databases like the National Technical Information Service, System for Information on Grey Literature in Europe-SIGLE, Current Controlled Trials, and the National Research Register (UK).

An attempt was done to contact each of the corresponding authors of the papers included in the study after thorough screening. This was done to avoid any type of omitted citations. Trials included in the study were on basis of type of grafting, postoperative rehabilitation, gender, surgery type, and case complexity. Papers were scrutinized on basis of relevancy of publication which was not a part of initial search strategy.

### 2.2. Exclusions Criteria

(1) Single case reports, incomplete datasets, guidelines, editorials, and review papers were excluded from the study. (2) Cases who were below 16 years of case were not considered in the study. (3) Incomplete details like where time range of surgery was not specifically mentioned were not included. (4) Papers mentioning ACL repair were excluded. (5) Non-English papers were excluded from the study. (6) Studies without any control group were excluded. (7) Full version of text missing was excluded. (8) Nonclear outcome was excluded.

RETRACTED

### 2.3. Inclusion Criteria

Investigators selected the articles on the basis of the inclusion criteria as follows: (1) patients with ACLR; (2) nonclear outcome was excluded; (3) reoperation rate, graft failure percentages, postoperative knee scores, complications in surgery, and outcomes reported; and (4) on the basis of study design: RCTs (randomized controlled trials) and non-RCTs.

### 2.4. Data Analysis and Statistical Assessment

Five meta-analyses were performed using RevMan 5.4.1 (as shown in Figure 2) (the Cochrane Collaboration, Copenhagen, Denmark): Graft Failure; Graft Diameter; IKDC score; Lysholm score; and Tegner Score. Continous variables were analyzed as mean ± SD. For the continuous variables, mean difference and 95% CI were evaluated.

## 3. Results

We analyzed six studies which met the inclusion criteria. The studies are mentioned and described in Table 1.

Graft failures are defined on the basis of post operation failures after a postoperative physical examination via either magnetic resonance imaging or anthroscopy. The ratio of failures of hybrid graft versus autograft was studied, and their characteristics are mentioned in Table 2. The odds ratio of hybrid graft versus autograft failures is analyzed using forest plot as shown in Figure 3, and funnel plotting of the same is shown in Figure 4.

Graft diameters are also an important factor to analyze the scenarios of graft failures; hence, they were compared and characteristics of hybrid graft versus autograft were analyzed which are shown in Table 3. The forest plot shows high heterogenicity of 95% CI 0.91 (0.65–1.18) in Figure 5, and the funnel plot for graft diameter of hybrid graft versus autograft is shown in Figure 6.

Abbreviations: CI, confidence interval; M-H, Mantel–Haenszel; the treatment of experimental group:hybrid graft. The control group:autograft. IKDC is a crucial parameter to analyze the level of knee injury in case of anterior cruciate ligament reconstruction; hence, it was compared for both hybrid graft and autograft, and the characteristics of both groups are shown in Table 4. The forest plot of the mean outcome differences in comparison of hybrid graft and autograft for International Knee Documentation Committee IKDC score is shown in Figure 7, and the funnel plot for the same is shown in Figure 8.

RETRACTED

Lysholm score of hybrid graft versus autograft plays another important parameter for analyzing the reconstruction surgery, and the characteristics of comparative analysis of both groups are shown in Table 5. The forest plot of the mean outcome differences in comparison of hybrid graft and autograft for International Knee Documentation Committee Lysholm score is shown in Figure 9, and the funnel plot for the same is shown in Figure 10.

Tegner score of hybrid graft versus autograft is compared for ACLR in hybrid graft and autograft groups as shown in Table 6. The forest plot of the mean outcome differences in comparison of hybrid graft and autograft for International Knee Documentation Committee Tenger score is shown in Figure 11, and the funnel plot is shown in Figure 12.

### 3.1. Limitations

First, aamples were small in most of the studies, so relatively large samples of Jacob and Leo et al. had a larger impact and influence in the results of meta-analysis. Second, many other potential factors affected the reconstruction surgery.

## 4. Discussion

In the past few years, allograft tendons have been used for augmenting the size of autograft in ACLR where good results were gained in comparison to allograft solely. The studies used for meta-analysis showed a similar kind of rate of success, performance failure, reoperation, revision, and retearing between hybrid graft and autograft patients.

In two studies out of the six, a slightly high IKDC scores and Lysholm scores were noted while comparing hybrid graft and autograft groups. Several studies have also shown a minor increase in failure rates post ACL reconstruction with soft tissues [16–18]. However, the benefits of increasing the graft diameter via hybrid graft over small diameter autograft have not been studied in much detail. The primary purpose of the study was to analyze the use of hybrid graft over autograft for ACL.

A lot of clinical trials have studied and supported the role of diameter in ACL. They have backed the use of ≥8 mm diameter of autograft in order to reduce the risk of ACLR revisions majorly for young people.

## 5. Conclusion

Most of the studies used have not shown any significant difference between hybrid graft and autograft studies. Studies mainly compare the outcome (patient-related), graft failures, measures of stability, and knee scores between the hybrid grafts and autografts groups.

## Figures and Tables

**Figure 1:** PRISMA flow diagram of the study selection process.

**Figure 2:** RevMan 5.4.1 was used to perform the statistical analysis.

**Figure 3:** Odds ratio of hybrid graft versus autograft failures. CI means confidence interval; M-H represents Mantel–Haenszel; the treatment of experimental group:hybrid graft. The control group:autograft.

RETRACTED

**Figure 4:** Funnel plot for failure of hybrid graft versus autograft; SE (log [RR]) means standard error via logarithmic transformation of relative risk.

**Figure 5:** Forest plot for graft diameter. CI means confidence interval; M-H represents Mantel–Haenszel; the treatment of experimental group:hybrid graft. The control group:autograft.

**Figure 6:** Funnel plot for graft diameter of hybrid graft versus autograft; SE (log [RR]) means standard error via logarithmic transformation of relative risk.

**Figure 7:** Forest plot for IKDC score of hybrid graft versus autograft.

**Figure 8:** Funnel plot for IKDC score of hybrid graft versus autograft.

**Figure 9:** Forest plot for Lysholm score of hybrid graft versus autograft. CI means confidence interval; M-H represents Mantel–Haenszel; the treatment of experimental group:hybrid graft. The control group:autograft.

**Figure 10:** Funnel plot Lysholm score of hybrid graft versus autograft.

**Figure 11:** Forest plot for Tegner score of hybrid graft versus autograft. CI means confidence interval; M-H represents Mantel–Haenszel; the treatment of experimental group:hybrid graft. The control group:autograft.

**Figure 12:** Funnel plot of Tegner score of hybrid graft versus autograft.

**Table 1:** Characteristics of ACLR included studies.

Criteria	[10]	[11]	[12]	[13]	[14]	[15]
**Study**						
Hybrid graft	42	37	31	24	29	28
Autograft	46	31	32	71	29	29

**Study design**	Cohort study	Prospective randomized controlled trial	Prospective randomized study	Retrospective comparative study	Retrospective comparative study	Retrospective comparative study

**Gender F/M**						
Hybrid graft	18/24	10/27	13/18	8/16	19/10	19/9
Autograft	26/20	15/16	15/17	25/46	19/10	19/10

**Duration of study**	From 2010 to 2015	From January 2014 to August 2017	From July 2005 to June 2008, China	February 2010 and April 2013	From 2007 to 2012	From July 2013 to July 2014

**Follow up**						
Hybrid graft	31.2	28.3	70.8	26.9	44.4	40.6
Autograft	46.7	28.4	69.6	26.9	48	40.6

**Graft diameter, mm**						
Hybrid graft	9.9 ± 0.8	8.3 ± 0.7	8 (NER)	Less than 8.5 mm (NER)	9.2 ± 0.9	9.1 ± 0.5
Autograft	7.8 ± 1.2	8.5 ± 0.7	8 (NER)	Less than 8.5 mm (NER	7.8 ± 0.7	8.8 ± 0.5

NER means not exact recorded.

**Table 2:** Ratio of failures of hybrid graft versus autograft.

Studies	Hybrid graft		Autograft	
	Events	Total	Events	Total
[14]	4	29	1	29
[10]	5	42	13	46
[13]	4	71	1	24
[15]	4	28	1	29
[11]	2	37	1	31

**Table 3:** Graft diameter (mm) used in hybrid graft versus autograft.

Studies	Hybrid graft			Autograft		
	Mean	SMD	Total	Mean	SMD	Total
[14]	9.2	0.9	29	7.8	0.7	29
[10]	9.9	0.8	42	7.8	1.2	46
[15]	9.1	0.5	28	8.8	0.5	29
[11]	8.3	0.7	37	8.5	0.7	31

RETRACTED

**Table 4:** IKDC score of hybrid graft versus autograft.

Studies	Hybrid graft			Autograft		
	Mean	S.D	Total	Mean	S.D	Total
[14]	71.3	19.5	29	86.1	13	29
[13]	89.3	4.6	24	87.3	7.4	71
[12]	89.8	5.7	31	87.5	3.2	32
[15]	71.6	6	28	75.7	4.6	29
[11]	85.9	4.8	37	84.7	6.7	31

**Table 5:** Lysholm score of hybrid graft versus autograft.

Studies	Hybrid graft			Autograft		
	Mean	S.D	Total	Mean	S.D	Total
[12]	90.5	10.2	31	91.3	11.5	32
[11]	89.2	5.4	37	88.3	6.5	31
[15]	81	10	28	89.6	4.7	29
[14]	80.2	12.2	29	90.3	11.2	29

**Table 6:** Tegner score of hybrid graft versus autograft.

Studies	Hybrid graft		Autograft			
	Mean	S.D	Total	Mean	S.D	Total
[12]	7.5	1.5	31	7.3	1.3	32
[15]	6.8	0.8	28	6.9	0.6	29
[11]	5.2	1.2	37	5.1	1.2	31

## Data Availability

The data used to support this study are obtained from the corresponding author upon request.
